# Effect of nicotinamide N-methyltransferase on lipid accumulation in 3T3-L1 adipocytes

This article has been retracted.

**DOI:** 10.1080/21655979.2022.2074768

**Published:** 2022-05-21

**Authors:** Wanfeng Xu, Ling Hou, Ping Li, Ling Li

**Affiliations:** a Department of Endocrinology, Shengjing Hospital of China Medical University, Shenyang, China; b Department of Pediatrics, Shengjing Hospital of China Medical University, Shenyang, China

**Keywords:** Nicotinamide N-methyltransferase, 3T3-L1 adipocytes, lipid accumulation, autophagy

## Abstract

Nicotinamide N-methyltransferase (NNMT) is a methylase, and its expression is positively correlated with obesity and insulin resistance. This study aims to detect the effects of NNMT on lipid accumulation, triglyceride content, adipocyte differentiation-related transcription factors, genes related to lipid metabolism, adipokine expression, and autophagy in adipocytes. Lentivirus vectors and eukaryotic expression plasmids were used to interfere with NNMT expression. The Oil Red O method was used to detect lipid accumulation, and colorimetry was used to detect triglyceride levels. The transcription of adipocyte differentiation-related transcription factors (PPARγ, C/EBPα, and SREBP1), lipid metabolism-related genes (*FABP4, FAS, FATP1* [*SLC27A1*], and *LPL*), adipokines (ADIPOQ and LEP) and autophagy-related genes (*Beclin1, ATG7, ATG12*, and *ATG14*) was detected by quantitative real-time polymerase chain reaction (RT-qPCR), and the protein expressions of PPARγ, ADIPOQ, LC3I, LC3II, Beclin1, and P62 were detected by western blot analysis. Compared with the control group, the knockdown of NNMT expression reduced lipid accumulation and triglyceride content in 3T3-L1 cells. The transcription of PPARγ, C/EBPα, SREBP1, *FABP4, FASN, FATP1, LPL, Beclin1, ATG7, ATG12*, and *ATG14* decreased, while ADIPOQ and LEP transcription increased. The expression of PPARγ, LC3I/II, and Beclin1 proteins also decreased, while ADIPOQ and P62 protein expression increased. The over-expression NNMT group showed experimental results opposite to those described above. Interference with the expression of NNMT affects lipid accumulation, triglyceride content after cell differentiation, adipocyte differentiation-related transcription factors, genes related to lipid metabolism, the expression of adipokines, and autophagy in adipocytes.

## Highlights

- This study found that knockdown of NNMT expression reduced lipid accumulation and triglyceride content in 3T3-L1 cells.
- Interference with the expression of NNMT also affects adipocyte differentiation-related transcription factors, genes related to lipid metabolism, the expression of adipokines, and autophagy in adipocytes.
- These results indicated that NNMT plays an essential role in these cellular processes.

## Introduction

Obesity has become a global issue, and its prevalence is increasing annually [1,2]. Worldwide, nearly 40% of adults have a body mass index higher than 25 kg/m^2^, and childhood obesity is rising in developed and developing countries [3]. Obesity is induced by an imbalance of energy intake and consumption and causes pathological lipid accumulation and adipocyte differentiation in the body, resulting in tissue dysfunction [4,5]. It is well known that it can cause insulin resistance, type 2 diabetes, heart disease, end-stage renal disease, and even some oncological diseases, seriously affecting patients’ quality of life [6]. Excessive accumulation of adipose tissue is suggested to be one of the leading causes of the aforementioned diseases [7]. Moreover, genetic data indicate that obesity may limit fat storage, resulting in insulin resistance [8]. Therefore, an in-depth study on the regulatory factors affecting adipose tissue accumulation is critical to improving this issue.

Adipose tissue is an endocrine organ and the main energy storage site in the human body. It secretes adipokines and hormones to maintain metabolic homeostasis [9]. When nutrient intake is excessive, white adipose tissue (WAT) is deposited to increase metabolic activity by inducing oxidative stress and a chronic low-grade inflammatory reaction before releasing free fatty acids (FFAs) into the plasma to regulate lipid metabolism [10,11].

Nicotinamide N-methyltransferase (NNMT) is an enzyme that methylates nicotinamide to form N1-methylnicotinamide, which can be discharged from the human body. The expression of NNMT in human adipose tissue is positively correlated with obesity and insulin resistance [12,13]. Studies have shown that NNMT expression knockdown can protect against lipid accumulation induced by a high-fat diet in C57BL/6 mice and significantly improve glucose tolerance compared with control groups [14]. Moreover, NNMT knockdown reduces body weight, fat mass, and insulin levels and improves glucose tolerance in female mice fed a Western diet, and has been shown to improve insulin sensitivity in male mice [15]. Neelakantan et al. used small-molecule NNMT inhibitors for the systemic treatment of diet-induced obese mice and found that they could significantly reduce body weight, WAT, adipose cell size, and plasma total cholesterol levels [16]. The mechanism includes the influence of SAM/NAD+ pathways and histone methylation. However, the effects and other mechanisms of NNMT on lipid accumulation in adipocytes remain unclear. Nicotinamide favored lipolysis in ovariectomized female rats [17], but the effects of NNMT on lipolysis remain unclear.

Autophagy is an essential physiological process that provides nutrients to maintain important cellular function in nutrient deficiency while removing excessive or damaged organelles and misfolded proteins and lipids in the state of nutrient overabundance. Studies have shown that the autophagy level of adipose tissue in obese patients is upregulated, and the lack of autophagy in adipose tissue inhibits the formation of lipid droplets, thereby inhibiting fat accumulation [18]. The influence of NNMT on autophagy remains unclear.

This study aimed to detect the effects of NNMT on lipid accumulation, triglyceride content, adipocyte differentiation-related transcription factors, genes related to lipid metabolism, adipokine expression, and autophagy in adipocytes. We hypothesized that NNMT played a vital role in these cellular processes.

## Materials and methods

### Cell culture

The 3T3-L1 cell line was purchased from the cell bank of the Chinese Academy of Sciences. The cells were cultured in Dulbecco’s Modified Eagle Medium (DMEM) high-glucose medium containing 10% calf serum in an incubator at a constant temperature of 37°C with 5% CO_2_ and sufficient humidity. After the cells grew 70%–80%, they were detached with 0.25% trypsin to form a single cell suspension passaged in a ratio of 1:2–1:3.

### The 3T3-L1 adipocyte induction differentiation program

The cells were inoculated into 6- or 12-well plates to achieve confluency of approximately 60% and then cultured (DMEM with 10% calf serum) for two days to 100% confluence. The cells were cultured for another two days (day 0) after the solution change. Next, they were cultured in induction solution I (DMEM containing 10% fetal bovine serum [FBS] with 0.5 mM IBMX, 1 μM dexamethasone, and 10 μg/ml insulin) for another two days (day 2) before being cultured in induction medium II (DMEM containing 10% FBS with 10 μg/ml insulin) for two days (day 4), followed by DMEM containing 10% FBS. The medium was changed once every two days (continuing for six days, eight days, etc.). The cells were collected for subsequent experiments according to the degree of cell induction and differentiation.

### The 3T3-L1 adipocyte Oil Red O staining step

The Oil Red O Kit (Solarbio, Beijing, China) was used to stain the 3T3-L1 adipocytes according to the manufacturer’s instructions. Differentiated and mature 3T3-L1 adipocytes were taken, fixed with 4% paraformaldehyde for 20 min after being washed, immersed in and washed with 60% isopropanol for 5 min, immersed in Oil Red O dye solution for 30 min, washed with deionized water (ddH_2_O) five times, and then photographed under a microscope. Next, 200 μL of isopropyl alcohol was added to each well; the cells oscillated on a shaker for 5 min. Finally, 200 μL of liquid was sucked into a 96-well plate and read at a 510 nm wavelength for the quantitative analysis.

### Vector construction and cell transfection

#### Design and synthesis of a mouse nicotinamide N-methyltransferase gene-targeted short hairpin RNA sequence

The NNMT gene sequence of mice (gene ID: 18113, NM_010924) was reviewed using the National Center for Biotechnology Information’s (NCBI) gene database. Three loci (Table 1) were selected using the Easy-siRNA design software, and two pairs of short hairpin RNA (shRNA) single-stranded oligonucleotide fragments (Genechem Co., Ltd., China) were designed and synthesized according to the shRNA design principles (Table 2).

**Table 1.** Easy-siRNA design

NO.	Accession	Target Seq	CDS	GC%
Nnmt-RNAi 1	NM_010924	gtCACCTATGTGTGTGATCTT	166.960	42.11%
Nnmt-RNAi 2	NM_010924	tgAGTCCTTCACGGAGATCAT	166.960	47.37%
Nnmt-RNAi 3	NM_010924	agAGTAGCTACTACATGATTG	166.960	36.84%
Description	Mus musculus nicotinamide N-methyltransferase (*Nnmt*), transcriptvariant 1, mRNA.

**Table 2.** Synthetic oligonucleotide information

NO.	5’	STEM	Loop	STEM	3’
Nnmt-RNAi 1-a	Ccgg	gtCACCTATGTGTGTGATCTT	CTCGAG	AAGATCACACACATAGGTGAC	TTTTTg
Nnmt-RNAi 1-b	aattcaaaaa	gtCACCTATGTGTGTGATCTT	CTCGAG	AAGATCACACACATAGGTGAC	
Nnmt-RNAi 2-a	Ccgg	tgAGTCCTTCACGGAGATCAT	CTCGAG	ATGATCTCCGTGAAGGACTCA	TTTTTg
Nnmt-RNAi 2-b	aattcaaaaa	tgAGTCCTTCACGGAGATCAT	CTCGAG	ATGATCTCCGTGAAGGACTCA	
Nnmt-RNAi 3-a	Ccgg	agAGTAGCTACTACATGATTG	CTCGAG	CAATCATGTAGTAGCTACTCT	TTTTTg
Nnmt-RNAi 3-b	aattcaaaaa	agAGTAGCTACTACATGATTG	CTCGAG	CAATCATGTAGTAGCTACTCT	

#### Construction of a mouse nicotinamide N-methyltransferase–short hairpin RNA fragment and lentivirus expression vector

A lentivirus expression vector with element sequence hU6-MCS-CBh-gcGFP-IRES-puromycin and control insertion sequence TTCTCCGAACGTGTCACGT was obtained from Genechem. The virus and double-stranded shRNA underwent double-enzyme digestion and were ligated overnight at 16°C using T4 DNA ligase. Following this, the exchange reaction products were transformed into competent cells cultured upside down in Luria-Bertani Petri dishes. Colonies were selected for polymerase chain reaction (PCR), sequencing, and identification. The prepared plasmid and virus packaging auxiliary plasmids, pHelper1.0 and pHelper2.0, were co-transduced into 293 T cells, and the supernatant was collected for concentration and titer determination after 48 h.

#### Transfection of nicotinamide N-methyltransferase lentivirus interference vector cells

The 3T3-L1 cells were inoculated into 24-well plates and grown in DMEM containing 10% calf serum when the cells grew up to 40%–50% in the plate within 24 h. Then, 20 μL of HiTransG P infection-boosting solution (Genechem) and 10 μL of NNMT lentivirus interference vector with a multiplicity of infection (MOI) of 100 or 10 μL of control vector were added to the cells after thorough mixing to achieve the required volume of 500 μL per well. The cell status was observed following overnight incubation, and the culture medium was replaced with fresh medium. Then, 48–72 h after infection, the expression of green fluorescent protein was observed under a fluorescence microscope. The downstream experiment was conducted if the fluorescence rate was greater than 80%. Finally, the cells were subcultured to induce differentiation for subsequent experiments.

#### Transfection of Nicotinamide N-methyltransferase overexpression plasmid cells

The 3T3-L1 cells were inoculated into 6-well plates and grown in DMEM containing 10% calf serum to achieve cell confluency of 80% at transfection. Next, 2 μg of the control plasmid and the NNMT overexpression plasmid (NCBI reference sequence: NM_010924.3, gene ID: 18113, synthesized by Changsha Youbao Bio) were added to 200 μL of jetPRIME buffer (Polyplus-transfection), vortexed for 10s, and then centrifuged. Following this, 4 μL of jetPRIME transfection reagent (Polyplus-transfection) was added, vortexed for one second, and incubated at room temperature for 10 min. This solution was then added to the cell culture medium. The culture medium was replaced with fresh medium every 24 h for subsequent experiments.

#### Triglyceride detection using a triglyceride colorimetric assay kit

A triglyceride colorimetric assay kit was obtained from Abbkine (China). According to the manufacturer’s instructions, 4 × 10^6^–5 × 10^6^ cells were collected, and 1 ml of extractive buffer was added to the cells. The cells were crushed by ultrasonic waves at 2 s intervals at 20% power for one minute. The samples were then centrifuged at 8,000 g for 10 min at 4°C, and the supernatant was taken. Next, 40 μL of supernatant, standard, and blank control (distilled and ddH_2_O) samples were collected, and 125 μL of extractive buffer was added to each sample and mixed thoroughly. Reagent I was added, shaken vigorously for 30s, and allowed to stand for 5 min; this process was repeated three times to obtain 15 μL of upper-layer solution. Then, 50 μL of reagent II and 15 μL of reagent III were added, and the mixture was treated in a water bath at 65°C for 3 min. Next, 50 μL of reagent IV and 50 μL of reagent V were added, and the mixture was treated in a water bath at 65°C for 15 min. After cooling, 100 μL of the medium was pipetted into a 96-well plate to determine the absorbance at 420 nm. The triglyceride content was measured using the calculation (measured value – blank value)/(standard – blank value), and the results were normalized for the protein concentration.

#### RNA extraction and real-time quantitative polymerase chain reaction

The cells were lysed with RNAiso Plus (Takara, Japan); the RNA was extracted according to the manufacturer’s instructions and then reverse-transcribed into complementary (cDNA) (Vazyme, China). Then, real-time quantitative PCR (RT-qPCR) was performed using the RT-qPCR kit SYBR Green Master Mix (Vazyme, China) and an RT-qPCR instrument (Roche, Shanghai, China). The reaction conditions were as follows: 95°C for 5 min, followed by 40 cycles at 95°C for 10s and 60°C for 30s, and then another stage at 95°C for 15s, 60°C for 60s, and 95°C for 15s. The data obtained from three independent experiments were analyzed using the formula RQ = 2^–ΔΔCt^. The primer sequences are detailed in Table 3.

**Table 3.** PCR primers list

GAPDH-Forward	5’-TTCAACGGCACAGTCAAGG-3’
GAPDH-Reverse	5’-CTCAGCACCAGCATCACC-3’
Fasn-Forward	5’-GGAGGTGGTGATAGCCGGTAT-3’
Fasn-Reverse	5’-TGGGTAATCCATAGAGCCCAG-3’
Slc27a1-Forward	5’-CGCTTTCTGCGTATCGTCTG-3’
Slc27a1-Reverse	5’-GATGCACGGGATCGTGTCT-3’
Fabp4-Forward	5’-AAGGTGAAGAGCATCATAACCCT-3’
Fabp4-Reverse	5’-TCACGCCTTTCATAACACATTCC-3’
Srebf1-Forward	5’-GATGTGCGAACTGGACACAG-3’
Srebf1-Reverse	5’-CATAGGGGGCGTCAAACAG-3’
Pparg-Forward	5’-GGAAGACCACTCGCATTCCTT-3’
Pparg-Reverse	5’-GTAATCAGCAACCATTGGGTCA-3’
Cebpa-Forward	5’-CAAGAACAGCAACGAGTACCG-3’
Cebpa-Reverse	5’-GTCACTGGTCAACTCCAGCAC-3’
Lpl-Forward	5’-GGGAGTTTGGCTCCAGAGTTT-3’
Lpl-Reverse	5’-TGTGTCTTCAGGGGTCCTTAG-3’
Adipoq-Forward	5’-TGTTCCTCTTAATCCTGCCCA-3’
Adipoq-Reverse	5’-CCAACCTGCACAAGTTCCCTT-3’
Lep-Forward	5’-GAGACCCCTGTGTCGGTTC-3’
Lep-Reverse	5’-CTGCGTGTGTGAAATGTCATTG-3’
Beclin1-Forward	5’-ACAGTGGACAGTTTGGCACA-3’
Beclin1-Reverse	5’-CGGCAGCTCCTTAGATTTGT-3’
ATG7-Forward	5’-TGCTATCCTGCCCTCTGTCTT-3’
ATG7-Reverse	5’-TGCCTCCTTTCTGGTTCTTTT-3’
ATG12-Forward	5’-CTTCTGGGCCTGCTGTTCACAGT-3’
ATG12-Reverse	5’-TTCTTGGGGTCAGCACAGACCTC-3’
ATG14-Forward	5’-ATCTTCTTGTGCAGTGCCAGCCTC-3’
ATG14-Reverse	5’-TTTGCCACTGCAAATGGCAGCC-3’

### Western blot analysis

The cells’ total protein content was extracted using RIPA lysis buffer (Beyotime, Shanghai, China), and the protein concentration (Thermo Fisher,Massachusetts, USA) was detected via the BCA method. The total protein loading was 20 μg; it was subjected to electrophoresis on 10% or 12.5% SDS-PAGE gel (Epizyme, Shanghai, China) and transferred to a 0.22 μm PVDF membrane (Millipore, Massachusetts, USA). It was incubated with 5% nonfat dried milk (blocking buffer) in the shaker for 1 h, and the primary antibody was incubated overnight at 4°C. The primary antibodies were anti-PPARγ (1:1,000, Cell Signaling Technology, Massachusetts, USA), anti-adiponectin (1:1,000, Cell Signaling Technology,Massachusetts, USA), ɑ-tubulin (1:3,000, ProteinTech, Chicago, USA), β-actin (1:300, Bioss, Beijing, China), GAPDH (1:300, Bioss, Beijing, China), anti-NNMT (1:500, 15123-1-AP, ProteinTech,Chicago, USA), anti-LC3 (1:1,000, Sigma,USA), Beclin 1 (1:1,000, Sigma, USA), and P62 (1:1,000, Sigma, USA). The secondary antibodies were diluted with PBST and incubated for 1 h at room temperature with goat anti-rabbit IgG horseradish peroxidase (1:3,000, Zsjqbio, Beijing, China) or goat anti-mouse IgG horseradish peroxidase (1:3,000, Zsjqbio, Beijing, China). The reactive bands were detected by an enhanced chemiluminescence kit (Tanon, Shanghai, China), after which the Image-Pro Plus gray-level analysis software was used to analyze the gray-level value of the displayed protein band. The sample’s relative expression was calculated using the expression of the internal reference protein as a control.

### Statistical analysis

The SPSS 18.0 software was used for the analysis, and the data were expressed as mean ± standard deviation. An analysis of variance or independent sample t-test was used to determine statistical differences, and P < 0.05 was considered statistically significant.

## Results

This study found that knockdown of NNMT expression reduced lipid accumulation and triglyceride content in 3T3-L1 cells. Meanwhile, the transcription of PPARγ, C/EBPα, SREBP1, *FABP4, FASN, FATP1, LPL, Beclin1, ATG7, ATG12*, and *ATG14* decreased, and ADIPOQ and LEP transcription increased. The expression of PPARγ, LC3I/II, and Beclin1 proteins also decreased, while ADIPOQ and P62 protein expression increased. The over-expression NNMT group showed experimental results opposite to those described above. These results indicated that NNMT played a vital role in these cellular processes.

### Nicotinamide N-methyltransferase and autophagy-related genes upregulated during 3T3-L1 cell differentiation

We detected the expression of NNMT and autophagy-related genes during the induction and differentiation of the 3T3-L1 cells (days 0, 2, 4, and 6). As shown in Figure 1, as the induction and differentiation time of the cells increased, the NNMT expression gradually increased (Figures 1(a,b)), as did the transcription of autophagy-related genes *Beclin1, ATG7, ATG12*, and *ATG14* (Figure 1(c)). The most significant increase in NNMT expression was observed on day 6, so we selected that day of 3T3-L1 cell differentiation induction for our follow-up experiments.

**Figure 1.** (a) Real-time quantitative polymerase chain reaction was used to detect the change of nicotinamide N-methyltransferase (NNMT) expression during 3T3-L1 cell differentiation, and NNMT mRNA expression was gradually increased on days 2, 4, and 6 of differentiation, especially on days 4 and 6 (****P < 0.0001), data represent mean ± standard deviation, and one-way analysis of variance was used for statistical analysis. (b) Western blot was used to detect the nicotinamide N-methyltransferase (NNMT) protein expression during 3T3-L1 cell differentiation. On days 2, 4, and 6 of differentiation, the NNMT protein increased gradually, especially on days 4 and 6 (*P < 0.05 and ***P < 0.001), data represent mean ± standard deviation, and one-way analysis of variance was used for statistical analysis. (c) Real-time qualitative polymerase chain reaction was used to detect the expression changes of autophagy-related genes Beclin1, ATG7, ATG12, and ATG14 during 3T3-L1 cell differentiation. With the gradual differentiation and maturation of the cells, autophagy was significantly increased, and the expression of autophagy-related genes was increased more significantly on day 6 (****P < 0.0001 and *P < 0.05), data represent mean ± standard deviation and one-way analysis of variance was used for statistical analysis.

### The knockdown expression of nicotinamide N-methyltransferase inhibited lipid accumulation during 3T3-L1 cell differentiation, accompanied by a decreased expression of transcription factors related to adipocyte differentiation and genes related to lipid metabolism, as well as increased adipokine expression

To further explore the effect of NNMT in differentiated 3T3-L1 adipocytes, we proceeded to knock down the expression of NNMT. When the cells’ MOI value was 100, the transfection efficiency reached more than 80%, and cell growth was strong (Figure 2(a)). Therefore, an MOI value of 100 was used in the follow-up experiments. LV-NNMT-RNAi was transduced into 3T3-L1 cells. Compared with the control group (LV-hU6-MCS-CBh-gcGFP-IRES-puromycin, control insertion sequence TTCTCCGAACGTGTCACGT), the NNMT messenger RNA (mRNA) levels and protein expression showed the most significant decrease in the LV-NNMT-RNAi3 group (Figures 2(b,c)), suggesting that the constructed LV-NNMT-RNAi3 lentivirus vector could effectively interfere with the expression of target protein NNMT in 3T3-L1 cells. Therefore, it was selected for subsequent experiments. Next, LV-NNMT-RNAi3 and the control virus vector were transduced into 3T3-L1 cells to induce differentiation. Compared with the control group, the lipid accumulation on day 6 of the induction and differentiation was significantly reduced in the LV-NNMT-RNAi3 group (Figures 2(d,e)), and the triglyceride content significantly decreased (Figure 2(f)). In order to explore the effect of NNMT on lipogenesis and lipolysis, we detected the transcription levels of adipocyte differentiation-related transcription factors, such as PPARγ, SREBP1, C/EBPα, and lipid metabolism-related genes, such as *FABP4, FASN, SLC27A1*, and *LPL*, significantly decreased, and the mRNA levels of adipokine ADIPOQ and LEP significantly increased (Figure 2(g)). Moreover, the protein expression of PPARγ was significantly reduced, while the protein expression of ADIPOQ significantly improved (Figure 2(h)).

**Figure 2.** (a) The lentivirus vector LV-Nnmt-RNAi, was transduced into 3T3-L1 cells at a multiplicity of infection value of 100, indicating that the transfection efficiency of the cells was above 80%. (b) The lentivirus vector LV-Nnmt-RNAi was transduced into 3T3-L1 cells, and a real-time quantitative polymerase chain reaction detected the changes of nicotinamide N-methyltransferase (NNMT) mRNA in 3T3-L1 cells. The expression of NNMT mRNA could be knocked down to 27% in the LV-Nnmt-RNA3 group compared with the control group (P < 0.0001), data represent mean ± standard deviation, and one-way analysis of variance was used for statistical significance analysis. (c) The lentivirus interference vector LV-Nnmt-RNAi was transduced into 3T3-L1 cells, and the expression of nicotinamide N-methyltransferase (NNMT) in 3T3-L1 cells was detected by western blot. The expression of NNMT protein could be knocked down to 19.5% in the LV-Nnmt-RNA3 group compared with the control group (P < 0.0001), data represent mean ± standard deviation, and one-way analysis of variance was used for statistical analysis. (d) Oil Red O staining was used to detect the lipid accumulation in 3T3-L1 cells on day 6 of induction and differentiation (40X, 100X, and 200X, respectively). Compared with the control group, the lipid accumulation in the LV-Nnmt-RNAi3 group was significantly reduced. Under the fluorescence microscope, it could be observed that GFP was still expressed after the induction and differentiation of 3T3-L1 cells, suggesting that the induction and differentiation process would not affect the effectiveness of the lentivirus interference vector. (e) The LV-Nnmt-RNAi3 and control groups were semi-quantitatively detected by Oil Red O staining (at 510 nm). Compared with the control group, the lipid accumulation in the nicotinamide N-methyltransferase (NNMT) knockout group was significantly decreased (1.000 ± 0.004 vs. 0.753 ± 0.008, P < 0.0001), data represent mean ± standard deviation, and a t-test was used for statistical analysis. (f) Compared with the control group, the triglyceride content in the LV-NNMT-RNAI3 group was significantly decreased on day 6 of induction and differentiation of 3T3-L1 cells (146.6 ± 14.02 vs. 73.16 ± 18.38 mg/mg protein, P < 0.05), data represent mean ± standard deviation, and a t-test was used for statistical analysis. (g) During the induction and differentiation of 3T3-L1 cells detected by real-time quantitative polymerase chain reaction, the mRNA levels of PPARγ, SREBF1, CEBPA, FABP4, FASN, SLC27A1, and LPL in the LV-NNMT-RNAI3 group were significantly decreased compared with the control group (on day 6). ADIPOQ and LEP mRNA were increased significantly (P < 0.0001), data represent mean ± standard deviation, and a t-test was used for statistical analysis. (h) During the induction and differentiation of 3T3-L1 cells detected by western blot, compared with the control group (on day 6), the expressions of nicotinamide N-methyltransferase (NNMT) and PPARγ proteins in the LV-Nnmt-RNAi3 group were significantly decreased (P < 0.0001) and the expression of adiponectin protein was significantly increased (P < 0.0001), data represent mean ± standard deviation, and a t-test was used for statistical analysis.

### The overexpression of nicotinamide N-methyltransferase promoted lipid accumulation during 3T3-L1 cell differentiation, accompanied by an increased expression of transcription factors related to adipocyte differentiation and genes related to lipid metabolism, as well as a decreased adipokine expression

Next, we overexpressed NNMT. The plasmid pcDNA3.1-NNMT-3xFlag-C was transduced into 3T3-L1 cells. Compared with the control group, the NNMT protein expression and mRNA levels were significantly increased in the transduced group (Figure 3(a,b)). The pcDNA3.1-NNMT-3xFlag-C plasmid and a control plasmid (pcDNA3.1–3xFlag-C) were then transduced into 3T3-L1 cells for induction and differentiation. Compared with the control group, the lipid accumulation on day 6 of the induction and differentiation was significantly increased in the cells transduced with pcDNA3.1-NNMT-3xFlag-C (Figure 3(c,d)). The triglyceride content also increased significantly (Figure 3(e)). In addition, the transcription levels of adipocyte differentiation-related transcription factors, such as PPARγ, SREBP1, C/EBPα, and lipid metabolism-related genes, such as *FABP4, FASN, SLC27A1*, and *LPL*, were significantly upregulated, while the mRNA levels of adipokine ADIPOQ and LEP were significantly downregulated (Figure 3(f)). The PPARγ protein expression was significantly decreased, while the ADIPOQ protein expression was significantly increased (Figure 3(g)).

**Figure 3.** (a) The pC DNA 3.1-NNMT-3xFlag-C plasmid was transduced into 3T3-L1 cells, and the transcriptional changes of nicotinamide N-methyltransferase (NNMT) mRNA in 3T3-L1 cells were detected by real-time quantitative polymerase chain reaction 24 hours after transfection. The results showed that the transcription of NNMT mRNA was significantly increased, which could be up to 5,655 times more than the control group (P < 0.0001). Data represent mean ± standard deviation, and a t-test was used for statistical analysis. (b) The pC DNA 3.1-NNMT-3xFlag-C plasmid was transduced into 3T3-L1 cells, and the expression changes of nicotinamide N-methyltransferase (NNMT) in 3T3-L1 cells were detected by western blot at 48 hours. The results showed that the expression of the NNMT over-expression group significantly increased, which could be up to 2.11 times more than the control group (P < 0.01). Data represent mean ± standard deviation, and a t-test was used for statistical analysis. (c) Oil Red O staining was used to detect the cell lipid accumulation on day 6 of induction and differentiation of 3T3-L1 cells (scale bar: 200 μm, 100 μm, 50 μm, respectively). Compared with the control group, lipid accumulation in the nicotinamide N-methyltransferase (NNMT) over-expression group was significantly increased. (d) The nicotinamide N-methyltransferase (NNMT) over-expression and control groups were semi-quantitatively detected by Oil Red O staining (at 510 nm). Compared with the control group, lipid accumulation in the NNMT over-expression group increased significantly (1.000 ± 0.032 vs. 1.467 ± 0.007, P < 0.0001). Data represent mean ± standard deviation, and a t-test was used for statistical analysis. (e) Compared with the control group, the triglyceride content in the nicotinamide N-methyltransferase (NNMT) over-expression group was significantly increased on day 6 of induction and differentiation of 3T3-L1 cells (117.2 ± 3.878 vs. 229.0 ± 4.704 mg/mg protein, P < 0.0001), data represent mean ± standard deviation and a t-test was used for statistical analysis. (f) During the induction and differentiation of 3T3-L1 cells detected by real-time quantitative polymerase chain, the mRNA level of PPARγ, SREBF1, CEBPA, FABP4, FASN, SLC27A1, and LPL in pcDNA3.1-NNMT-3xFlag-C over-expression group was significantly increased compared with the control group (on day 6). ADIPOQ and LEP mRNA was significantly decreased (P < 0.0001), data represent mean ± standard deviation, and a t-test was used for statistical analysis. (g) During the induction and differentiation of 3T3-L1 cells detected by western blot, compared with the control group (on day 6), the expression of nicotinamide N-methyltransferase (NNMT) and PPARγ proteins in the pcDNA3.1-NNMT-3xFlag plasmid group were significantly increased (P < 0.0001) and the expression of adiponectin protein was significantly decreased (P < 0.0001), data represent mean ± standard deviation, and a t-test was used for statistical analysis.

### Interference with the expression of nicotinamide N-methyltransferase can change the autophagy-related genes during 3T3-L1 cell induction and differentiation

As mentioned previously, we found that the NNMT and autophagy-related genes increased during the induction and differentiation of the 3T3-L1 cells. To investigate whether NNMT could influence autophagy-related genes in 3T3-L1 cells, LV-NNMT-RNAi3 and pcDNA3.1-NNMT-3xFlag-C were transduced into the cells and induced to differentiate. The change in the autophagy-related genes on day 6 was recorded. Compared with the control group, the knockdown of NNMT expression resulted in a significant decrease in the mRNA levels of *Beclin1, ATG7, ATG12*, and *ATG14* (Figure 4(a)). In addition, the protein expression of LC3I/II and Beclin 1 significantly decreased, and the P62 protein level significantly increased (Figure 4(b)). LC3 is processed by ATG4 to reveal an LC3-I, then the ATG12–ATG5-ATG16L1 complex participates in the conjugation of PE to LC3-I to create LC3-II, which associates with the phagophore in autophagy. So the LC3I/II ratio might be an indicator of autophagic flux. Conversely, in the overexpression NNMT group, the mRNA levels of *Beclin1, ATG7, ATG12*, and *ATG14* significantly increased (Figure 4(c)), the protein expression of LC3I/II and Beclin1 significantly increased, and the P62 protein level significantly decreased (Figure 4(d)). These results suggested that interference with NNMT expression in 3T3-L1 cells could change the autophagy level during differentiation induction.

**Figure 4.** (a) During the induction and differentiation of 3T3-L1 cells detected by real-time quantitative polymerase chain, compared with the control group (on day 6), the mRNA levels of Beclin1, ATG7, ATG12, and ATG 14 in the LV-NNMT-RNAI3 group were significantly decreased (P < 0.0001, P < 0.01, P < 0.05). Data represent mean ± standard deviation, and a one-way analysis of variance was used for statistical analysis. (b) During the induction and differentiation of 3T3-L1 cells detected by western blot, compared with the control group (on day 6), the LC3 II/I ratio and Beclin 1 protein expression were significantly decreased, and P62 protein was significantly increased in the LV-Nnmt-RNAi3 group (P < 0.0001). Data represent mean ± standard deviation, and a t-test was used for statistical analysis. (c) During the induction and differentiation of 3T3-L1 cells detected by real-time quantitative polymerase chain, compared with the control group (on day 6), the mRNA levels of Beclin1, ATG7, ATG12, and ATG 14 in the pcDNA3.1-Nnmt-3xFlag-C over-expression group was significantly increased (P < 0.0001, P < 0.05). Data represent mean ± standard deviation, and a one-way analysis of variance was used for statistical analysis. (d) During the induction and differentiation of 3T3-L1 cells detected by western blot, compared with the control group (on day 6), the LC3 II/I ratio and Beclin 1 protein expression of pcDNA3.1-NNMT-3XFlag-c over-expression group were significantly increased, while the P62 protein was significantly decreased (P < 0.0001). Data represent mean ± standard deviation, and a t-test was used for statistical analysis.

## Discussion

The rising prevalence of obesity is a global health issue that leads to an increased risk of disease [19]. According to Keaver et al., by 2030, 89% of men and 85% of women in Ireland will be categorized as overweight or obese, which will lead to a 97% increase in the incidence of obesity-related coronary heart disease, a 61% increase in cancer, and a 21% increase in type 2 diabetes [20]. There are also economic implications. Hayes et al. found that the medical cost for obese children was 1.62 times that of children of normal weight in Australia [21].

The differentiation and lipid accumulation of adipocytes are closely related to the occurrence and development of obesity [22]. In a study of obese mice, NNMT knockdown reduced body weight, fat loss, and insulin levels, thereby improving glucose tolerance. It may be that NNMT knockdown increased the ratio of SAM/SAH and overall histone H3K4 methylation, which was related to transcriptional activation. Various studies have also shown that the level of autophagy in the adipose tissues of obese human patients and mice is significantly increased [22,23] and that autophagy inhibition can reduce obesity [23]. Singh and his colleague found that knockdown of *Atg7* in 3T3-L1 preadipocytes inhibits lipid accumulation and decreases the protein levels of adipocyte differentiation factors [24]. Knockdown of *Atg5* or pharmacological inhibition of autophagy had similar effects [24]. An adipocyte-specific mouse knockout of *Atg7* generated lean mice with decreased WAT mass and enhanced insulin sensitivity [24]. Some studies found NNMT related to autophagy [25–29]. Shin et al. found that NNMT could be a negative autophagy regulator in liver cancer [25]. Nicotinamide N-methyltransferase inhibits the autophagy induced by oxidative stress in breast cancer cells [26]. High neuronal ANMT-1 (the nematode NNMT ortholog) activity induces autophagy via the NPRL-2/NPRL2 pathway [27]. Both bafilomycin A1 and chloroquine abrogated the increase in NNMT expression caused by glucose deprivation, suggesting that autophagy is involved in regulating NNMT expression [28,29]. In this study, we found that during the differentiation of 3T3-L1 cells to mature adipocytes, the NNMT expression and the autophagy level gradually increased. This increase was most significant on the sixth day. Therefore, we speculated that NNMT might participate in obesity regulation through autophagy.

The effect of NNMT on adipocyte differentiation-related transcription factors PPARγ, C/EBPα, and SREBP1 was explored in this study. A ligand-activated transcription factor, PPARγ’s expression is highest in adipocytes, plays a key role in lipogenesis, energy balance, and lipid biosynthesis, and is also involved in lipoprotein metabolism and insulin sensitivity [30,31]. Consistent with this information, we found that interference with NNMT expression during the induction and differentiation of the 3T3-L1 cells caused changes in the PPARγ expression and affected the corresponding lipid accumulation and triglyceride content.

Highly conservative members of the basic leucine zipper protein family, C/EBPα, are an important transcription factor involved in regulating adipogenic differentiation. Research has shown that C/EBPα knockout mice display metabolic abnormalities and cannot complete lipid accumulation in the adipocytes [32]. A transcription factor with a spiral-loop-spiral leucine zipper domain, SREBP1 is involved in regulating adipocyte differentiation by controlling the expression of genes related to the synthesis and uptake of cholesterol, fatty acids, and triglycerides [33]. In this study, we found that interference with NNMT expression caused a change in the transcription levels of C/EBPα and SREBP1 during the 3T3-L1 cell differentiation.

We also explored the effect of NNMT on lipid metabolism-related genes *FABP4, FASN, SLC27A1*, and *LPL* and adipokines ADIPOQ and LEP. As one of the most abundant proteins in adipocytes, through interaction with hormone-sensitive lipase and PPARγ, FABP4 maintains lipocyte homeostasis and regulates lipolysis and lipogenesis [34]. Genetic disruption of FABP4 in obese mice causes a significant decrease in plasma insulin, glucose, triglyceride, and cholesterol levels [35]. A key enzyme regulating the *de novo* synthesis of intracellular fatty acids, FASN can catalyze the synthesis of long-chain fatty acids from acetyl-CoA [36]. As one of the fatty acid transporter families, *SLC27A1* is involved in the uptake and metabolism of long-chain fatty acids. Studies have shown that after the knockout of the *SLC27A1* gene in mice, the fatty acid uptake in the adipocytes decreases significantly; thus, it can control diet-induced obesity and insulin resistance [37]. Next, LPL is a member of the triacylglycerol esterase family. Researchers have shown that during preadipocyte differentiation, the expression of LPL increases significantly with the accumulation of triglycerides. Therefore, it has been suggested that LPL is an important gene marking adipocyte differentiation [38]. A protein factor specifically secreted by adipocytes, ADIPOQ can regulate insulin sensitivity and energy balance and reduce glucose, fatty acid, and triglyceride levels. Finally, LEP reduces lipid accumulation in adipocytes by increasing triglyceride turnover, inhibiting the re-synthesis of fatty acids, and stimulating the oxidation of glucose and FFAs [39]. We found that during the induction and differentiation of 3T3-L1 cells, interference with NNMT expression leads to changes in the transcriptional activities of fat metabolism-related genes *FABP4, FASN, SLC27A1*, and *LPL*, thereby affecting lipid accumulation. Moreover, it results in changes in the transcriptional activities of adipokines ADIPOQ and LEP, which also affects lipid accumulation.

To investigate the effects of NNMT on adipocyte function and the possible mechanisms of its action, we used lentiviral knockdown and overexpression plasmids to interfere with – and then induce – differentiation. On day 6, we observed a significantly decreased number of cells with lipids. Smaller and fewer lipid droplets formed in the 3T3-L1 cells, decreasing the fat accumulation and triglyceride content in the NNMT knockout group. Moreover, the transcription of adipocyte differentiation-related transcription factors PPARγ, C/EBPα, and SREBP1 decreased, as did the expression of PPARγ protein. The transcription of the *FABP4, FASN, FATP1*, and *LPL* genes related to lipid metabolism were downregulated, while the transcription of ADIPOQ and LEP and the expression of the ADIPOQ protein increased. Therefore, we believe that NNMT may regulate the expression of these genes in lipid accumulation. In addition, the transcription of autophagy-related genes *Beclin1, ATG7, ATG12*, and *ATG14* was decreased along with the protein expression ratio of LC3II/I and the protein expression of Beclin 1. Moreover, the increased expression of P62 compared with the control group indicated reduced levels of autophagy. Thus, we think that the mechanism of NNMT in lipid accumulation may also include autophagy regulation. An inverse result was observed in the overexpression NNMT group. The above results indicated that interference with NNMT affects lipid accumulation in 3T3-L1 cells, possibly by interfering with the transcription and expression of PPARγ, C/EBPα, and SREBP1 and affecting the functions of FABP4, FAS, FATP1, and LPL, which might be related to autophagy.

N1-methylnicotinamide, a metabolite of NNMT, was found to be able to inhibit reactive oxygen species, inflammation, apoptosis in palmitic acid-treated H9C2 cells and improve inflammation, apoptosis, and fibrosis damage in free fatty acids-bound-albumin-overloaded mice. [40] In our study, knockdown of the expression of NNMT could ameliorate the lipid accumulation in adipocytes, maybe due to the knockdown of NNMT causing the increase of N1-methylnicotinamide, which inhibits reactive oxygen species.

This study had some limitations. First, we didn’t analyze the potential influence of different genders. Furthermore, the effect of NNMT inhibition in fully differentiated cells was also not investigated. Future studies would focus on the effects of N1-methylnicotinamide and the substrate of NNMT on adipocytes. Whether the obese phenotype was able to be reversed when adipocytes were already present and loaded with lipids also deserves to be investigated.

## Conclusion

In conclusion, knockdown of NNMT expression reduced lipid accumulation and triglyceride content in 3T3-L1 cells. Meanwhile, the transcription of PPARγ, C/EBPα, SREBP1, *FABP4, FASN, FATP1, LPL, Beclin1, ATG7, ATG12*, and *ATG14* decreased, and ADIPOQ and LEP transcription increased. The expression of PPARγ, LC3I/II, and Beclin1 proteins also decreased, while ADIPOQ and P62 protein expression increased. The over-expression NNMT group showed experimental results opposite to those described above. These results indicated that NNMT played an essential role in these cellular processes.
